# MiR-130a-3p suppresses colorectal cancer growth by targeting Wnt Family Member 1 (WNT1)

**DOI:** 10.1080/21655979.2021.1977556

**Published:** 2021-10-18

**Authors:** Guang-Lin Song, Ming Xiao, Xiao-Ya Wan, Jun Deng, Jun-Da Ling, Ying-Guo Tian, Min Li, Jie Yin, Ren-Ying Zheng, Yi Tang, Gui-Yuan Liu

**Affiliations:** a Department of Oncology, People’s Hospital of Yuechi County, Yuechi County, Sichuan Province, China; b Department of Pathology, Molecular Medicine and Cancer Research Center, Chongqing Medical University, Chongqing, China; c Department of General Surgery, The Affiliated Hospital of Chongqing Three Gorges, Chongqing, China

**Keywords:** Colorectal cancer, miR-130a-3p, tumor suppression, WNT1, Wnt signaling pathway

## Abstract

The microRNA miR-130a-3p (miR-130a-3p) has anti-tumor activity against numerous cancer types. Further, miR-130a-3p may target Wnt signaling, which is a critical pathway regulating tumorigenesis. Functions of miR-130a-3p in colorectal cancer (CRC) and contributions of Wnt1 pathway modulation, however, have not been examined, hence the exploration on these two aspects. In this study, in comparison with normal controls, both CRC tissue and multiple CRC cell lines showed downregulated miR-130a-3p. MiR-130a-3p overexpression contributed to a decrease in CRC cell proliferation. Additionally, its overexpression also caused reduced expression of WNT Family Member 1 (WNT1) and downstream WNT pathway factors c-myc and cyclin D1. Dual-luciferase assay revealed WNT1 as a direct target of miR-130a-3p, and further the inhibitory effect of miR-130a-3p on c-myc and cyclin D1 was proved to be reversed by overexpressed WNT1. Collectively, miR-130a-3p inhibits CRC growth by directly targeting WNT1, and miR-130a-3p and WNT1 pathway-associated factors are defined as potential targets for CRC treatment.

## Introduction

Colorectal cancer (CRC) is one of the tumors contributing the most to the incidence among malignancies. According to data released by the American Cancer Society in 2018, the annual global incidence of CRC is 1.8 million, accounting for 10.2% of the total and ranking third; its mortality accounts for 9.2% of the total and ranks second [1]. The American Joint Committee on Cancer staging is currently the most widely used staging method for CRC, and a 5-year overall survival decreases progressively from 90% to less than 10% from stage I to stage IV [2,3]. While survival has risen due to improvements in surgery, radiotherapy, chemotherapy, targeted therapy, and other treatments, the prognosis for advanced-stage CRC is still poor. Therefore, new treatment methods and therapeutic targets are required to improve CRC survival.

MicroRNAs (miRNAs) are endogenous small non-coding RNA molecules containing about 22 nucleotides expressed widely among animals, plants, and even some viruses [4]. Numerous studies have reported abnormal expression of miRNAs in tumors, and some have directly implicated aberrant expression in tumorigenesis and progression [5–7]. Iida et al. found that overexpression of miRNA-221/222 can promote the proliferation and metastasis of various cancer cells and suppress apoptosis [8]. Takamizawa and colleagues first reported that let-7 expression is often reduced in lung cancer [9], and Li et al. reported that miRNA-551a and miRNA-495 inhibit expression of the carcinogenic factor PRL-3-UTR and also suppress gastric cancer cell invasion and metastasis [10]. MiR-130a-3p affects multiple tumor progression and miR-130a is located on chromosome 11q12.1 in the intron of gene AP000662.4 [11]. Specifically, the suppression of invasion and metastasis of breast cancer stem cell-like cells by miR-130a-3p was achieved through targeting RAB5B [12], and the inhibition of proliferation, invasion, and metastasis of nasopharyngeal carcinoma (NPC) cells by this miRNA was achieved by inhibiting the expression of BACH2 [13] and CXCL12 [14]. Further, in the study by Wang et al., miR-130a-3p caused lower TBL1XR1 expression and inhibition of the mesenchymal transformation, invasion, and metastasis of gastric cancer epithelial cells [15]. These studies have showed miR-130a-3p negatively affecting various cancer development. According to recent studies, miR-130a-3p is also expressed in CRC. Kara et al. [16] screened by high-throughput sequencing and found a significant down-regulation of miR-301a-3p CRC tumor tissues. However, no studies were searched on what miR-130a-3p affected CRC or on potential targets. In addition, human CRC tissues showed lowly expressed miR-130a-3p in comparison with normal tissues from the Cancer Genome Atlas (TCGA) database. Wnt Family Member 1 (WNT1) is a member of the Wnt family. Dysregulated Wnt signaling is implicated in the development of colon cancer and breast cancer among other [17]. It has been reported that Wnt1 is the downstream target for miRNAs [18]. Therefore, *in vivo and in intro* experiments were conducted to determine what and how miR-130a-3p regulated CRC progression via the target WNT1, thereby providing potential novel therapeutic targets and biomarkers for CRC.

## Materials and methods

### Tissue samples

Thirty CRC and adjacent tissue samples were acquired via General Surgery Department of the Affiliated Hospital of Chongqing Three Gorges Medical College from February 2018 to August 2018. Specimen retrieval was approved by all patients and by the institutional ethics committee. Samples were stored in liquid nitrogen until analyses.

### Data collection

CRC datasets were downloaded from the Cancer Genome Atlas (TCGA) data portal (http://tcga-data.nci.nih.gov) and gene expression evaluated in the TCGA RNA-Seq dataset. The relationship between miR-130a-3p with tumorigenesis and prognostic value was analyzed using survival data obtained from TCGA that were submitted to online analysis tool Oncomir (http://www.oncomir.org/) and OncoLnc (http://www.oncolnc.org/).

### Cell culture and cell transfection

After being purchased from Shanghai Cell Bank of Chinese Academy of Sciences (China), human CRC cell lines SW480, LOVO, HCT116, SW620, and HT29 and the normal colon epithelial cell line NCM460 were then maintained in RPMI-1640 medium with supplement of 100 IU/ml streptomycin (Hyclone, Logan, UT, USA), 100 IU/ml penicillin, 10% fetal bovine serum (FBS, Hangzhou Sijiqing Company, China). The culture conditions were as follows: a humidified atmosphere containing 5% CO_2_ at 37°C.

MiR-130a-3p mimics (5ʹ-CAGUGCAAUGUUAAAAGGGCAU-3ʹ), from Shanghai GenePharma Co., Ltd (China), were transfected into HCT116 and SW480 cells according to the instruction of Lipofectamine 2000 (Invitrogen, Carlsbad, CA, USA). Mimic negative control (5ʹ-CAGUACUUUUGUGUAGUACAA-3ʹ) was also provided by the same company.

### Real time quantitative PCR (RT-qPCR)

Following the extraction of total RNA by TRIzol reagent (Invitrogen, USA), reverse transcription was conducted in accordance with the TaqMan@MicroRNA reverse transcription kit instruction (Takara, Japan). Subsequently, RT-qPCR was performed using a qPCR kit (Takara, Japan), with primers, shown in Table 1, synthesized by Sangon Biotech Co. (Shanghai, China) (Table 1). Each experiment was performed in triplicate.

**Table 1.** Primer sequences for RT-qPCR

Gene	Sequence (5ʹ-3ʹ)	
miR-130a-3p	TGCTGCTGGC CAGAGCTCTT	CACTACACGGCCAATGCCC
wnt1	AGGTTCCATCGAATCCTGCAC	CATCTCGGAGAATACGGTCGT
c-myc	GGCTCCTGGCAAAAGGTCA	CTGCGTAGTTGTGCTGATGT
cyclin D1	CAATGACCCCGCACGATTTC	CATGGAGGGCGGATTGGAA
U6	CTCGCTTCG GCAGCACA	AACGCTTCACGAATTTGCGT

*Western blotting* Protein extraction protocols (Beyotime, Shanghai, China) were obeyed to extract total protein from cells or tissues, followed by concentration determined by a BCA assay (Beyotime). Proteins were mixed with 5× protein buffer at 4:1 and denatured in boiling water for 10 min. The protein samples were then separated at 30–50 μg per gel lane by SDS-PAGE electrophoresis using the following settings: 80 V, 250 mA constant current, and 1 h at room temperature. Proteins were then electrotransferred to PVDF membranes, followed by blocking step using 5% skimmed milk powder. Subsequently, an overnight incubation of the membranes was carried out at 4°C in Tris-buffered saline plus 1% Triton-X (TBST) containing anti-β-actin (1:1000, the gel-loading control), anti-WNT1 (1:500), anti-cyclin D1 (1:500), and (or) anti-c-myc (1:500) (all from Proteintech, Chicago, IL, USA). Next, the membranes were rinsed with TBST (10 min/time, totally 3 times), incubated in peroxidase-conjugated goat anti-rabbit IgG (Boster, Wuhan, China) for 2 h, and rinsed three times using TBST (5 min/time). Immunolabeling was visualized using a chemiluminescence imager and expression quantified as the grayscale value of the target band to the β-actin band. Each experiment was repeated three times.

### Dual-Luciferase reporter assay

The putative targeting gene WNT1 of miR-130a-3p was predicted using miRwalk (http://www.ma.uni-heidelberg.de/apps/zmf/miRwalk/), miRanda (http://www.miRanda-im.org/) and TargetScan (http://www.targetscan.org/). WNT1 3ʹ-UTR (WNT1-WT, containing the putative binding site of miR-130a-3p) and mutant WNT1 3ʹ-UTR (WNT1-MUT) were cloned into the pGL3-basic vector (Promega, Madison, WI, USA). Next, co-transfection of miR-130a-3p mimics or negative control and WNT1-WT or WNT1-MUT into HEK-293 T cells was achieved by utilizing Lipofectamine 2000. On completion of measurement of firefly (hLuc) and Renilla (hRluc) luciferase activities by a fluorescence illuminometer, the fluorescence values of hRluc were compared with those of hLuc, and the ratios of transfected cells to controls were analyzed.

### Colony formation assay

Cells from each transfection group (miR-130a-3p mimics, mimics control, untransfected control) were plated at 100 cells per well with six replicates. After 14 days in culture, cells were washed and fixed with methanol for a period of 30 min. On completion of the 30-min fixation, 0.4% crystal violet was adopted for staining for a period of 15 min. Finally, colonies formed in each transfection group were counted.

*CCK-8 assay*. CCK-8 (Dojindo, Shanghai, China) was added at 24, 48, and 72 h after transfection, followed by 2 h cell culture at 37**°**C. Finally, measurement of the optical density (OD450) was carried out, and the value was as an estimate of viable cell number.

### Subcutaneous tumorigenesis in nude mice

Female SPF BALB/c nude mice aged 6–8 weeks were housed and then grouped into miR-130a-3p mimic, mimic control, and Control groups (6 mice/group). For the tumor formation experiment, transfected HCT116 or SW480 (5 × 10^6^ cells) were subcutaneously injected into the right flank of each mouse. The mice were sacrificed for excising tumor tissues after 40 days, and tumor length, width, and volume (volume = 0.5 × length × width^2^) were measured for each group.

### Statistical analysis

Data were statistically analyzed by using SPSS 20.0 software, and finally expressed in mean ± standard deviation (SD). Differences between or among groups were compared by utilizing one-way ANOVA or Student’s t-test. A significant difference was indicated if P < 0.05 (two-tailed).

## Results

### MiR-130a-3p is underexpressed in colorectal cancer

We first analyzed the clinical samples from the TCGA database and found lower miR-130a-3p expression in comparison with normal colon tissues (Figure 1a-b). To provide further evidence for reduced miR-130a-3p expression in CRC, we measured the expression in CRC tissues, paracarcinoma tissue, and cultured cells by RT-qPCR. Consistent with the TCGA database, miR-130a-3p expression was significantly lower in CRC tissues than in corresponding paracarcinoma tissue (Figure 1c-d). Similarly, multiple CRC cells lines (HCT116, SW480, LOVO, SW620, and HT29) exhibited a markedly decreased miR-130a-3p expression in comparison with the noncancerous colon mucosal epithelial cell line NCM460 (Figure 1e). In colon carcinoma, Kaplan–Meier survival curves and log-rank test to evaluate the prognostic value of miR-130a-3p. The result showed that the CRC patients with low level of miR-130a-3p had a worse survival (figure 1f). MiR-130a-3p also has associated with tumorigenesis of CRC (Figure 1g).

**Figure 1.** Downregulation of miR-130a-3p expression in colorectal cancer tissue and cell lines, and the linkage between miR-130a-3p and colon carcinoma. (a, b) miR-130a-3p expression in CRC samples and normal tissue from the TCGA database. (c, d) miR-130a-3p expression in CRC tissue samples versus adjacent noncancerous tissue. (e) Comparison of miR-130a-3p expression among multiple CRC cell lines and a noncancerous colon epithelial cell line. Expression levels in (c–e) were estimated by RT-qPCR. (f) Kaplan-Meier survival curves are used to evaluate the prognostic value of miR-130a-3p in CRC. (g) miR-130a-3p has significantly associated with tumorigenesis of CRC. CRC, colorectal cancer. *P < 0.05, ** P < 0.01

### MiR-130a-3p overexpression inhibits colorectal cancer cell proliferation

After SW480 and HCT116 cells were transfected miR-130a-3p mimics, the RT-qPCR has been shown that the expression of miR-130a-3p was increased, compared with control groups (Figure 2a-b). To directly examine what effects miR-130a-3p had on CRC cell tumorigenic properties, a comparison was carried out among HCT116 and SW480 cells after transfecting miR-130a-3p mimics or mimics control. As measured by CCK-8, in overexpressed miR-130a-3p significantly reduced CRC cell viability compared to the corresponding untransfected control and mimics control (Figure 2c-d). Similarly, overexpressed miR-130a-3p decreased CRC cell colony formation (Figure 2e-f).

**Figure 2.** MiR-130a-3p overexpression inhibits CRC cell proliferation. (a, b) The miR-130a-3p level was increased in miR-120a-3p transfected SW480 and HCT116 cells. (c, d) CCK-8 assay for examining CRC cell viability. (e, f) Results of CRC cell colony formation assay. CRC, colorectal cancer. **P < 0.01

### WNT1 is a direct downstream target of miR-130a-3p

TargetScan, RIRDB, and RIWALK programs identified that WNT1 was potentially a downstream target of miR-130a-3p. In colorectal carcinoma tissues, the results of RT-qPCR also showed that the expression of WNT1 mRNA was increased, compared with normal colon tissues (Figure 3a). Subsequently, RT-qPCR-based and western blot-based assays were performed for comparing WNT1 mRNA and protein expression, aiming to determine if miR-130a-3p targets WNT1 mRNA for degradation. Consistent with WNT1 targeting, both mRNA and protein levels were significantly lower in HCT116 and SW480 cells in the miR-130a-3p mimics group compared with the mimics control (Figure 3b-e). To examine whether WNT1 downregulation was due to direct binding with the miRNA, we then conducted luciferase expression assays for comparing WNT1 expression between CRC cells expressing the wild-type 3ʹ-UTR sequence of WNT1 or a sequence mutated within the putative binding region (figure 3f). Consistent with direct binding, co-transfection of wild-type WNT1 with miR-130a-3p mimics led to a marked decrease in luciferase activity (P < 0.01), suggesting that miR-130a-3p mimics reduced wild-type WNT1 expression; the co-transfection of mut1 or mut2 WNT1 3ʹ-UTR with miR-130a-3p mimics was also associated with a decline in luciferase activity, but the degree of decline was not as significant as that of the whole wild type group (P < 0.05), whereas two binding sites mutate together had no effect on luciferase activity. (Figure 3g) Therefore, it is suggested that WNT1 is a direct downstream target of miR-130a-3p.

**Figure 3.** WNT1 is a direct target gene of miR-130a-3p. (a) RT-qPCR was used to detect the WNT1 mRNA expression in human CRC tissues and normal colon tissues. (b, c) Quantitation of WNT1 protein by western blot in untreated CRC cells (Control) and CRC cells with transfection of mimics control or miR-130a-3p mimics. (d, e) RT-qPCR for determining expression of WNT1 mRNA in SW480 and HCT116 cell. WNT1 expression was reduced at both protein and mRNA levels by miR-130a-3p overexpression. (f) Sequence diagrams of wild-type WNT1 3ʹ-UTR, corresponding mutant WNT1 3ʹ-UTR, and miR-130a-3p showing putative complementary binding sites. (g) Reporter assay showing that only wild-type WNT1 3ʹ-UTR suppressed luciferase activity. CRC, colorectal cancer. *P < 0.05 and **P < 0.01 vs controls

### MiR-130a-3p overexpression reduces cyclin D1 and c-myc expression

Cyclin D1 and c-myc are downstream targets of the WNT pathway. The results of RT-qPCR showed that the expression of cyclin D1 and c-myc mRNA was increased in colorectal carcinoma tissues compared with normal colon tissues (Figure 4 A-B). And then, miR-130a-3p mimics transfection was to prove that overexpressed miR-130a-3p downregulated expression levels of WNT signaling targets cyclin D1 and c-myc in SW480 and HCT116 cells, comparison with the control groups (Figure 4 C-J).

**Figure 4.** Downregulation of cyclin D1 and c-myc by miR-130a-3p overexpression. (a-b) RT-qPCR was performed to measure the mRNA expression of cyclin D1 and c-myc in human CRC tissues and normal colon tissues. (c-f) Western blotting for determining Cyclin D1 and c-myc protein expression in control, mimic control, and mimic transfection CRC cell groups. (g-j) RT-qPCR results. Reduction of cyclin D1 and c-myc in CRC cell lines by miR-130a-3p overexpression (mimics group), compared with control and mimics control groups. CRC, colorectal cancer. *P < 0.05, **P < 0.01

### WNT1 overexpression reduces the suppressive effect of miR-130a-3p on c-myc and cyclin D1

Furthermore, we performed cell rescue experiments. The reduction in cyclin D1 and c-myc levels induced by miR-130a-3p overexpression in CRC cells were reversed by co-transfection of a WNT1 overexpression vector (pHAHE+WNT1) (Figure 5a-f). In addition, overexpression of WNT1 also achieved the reversal of downregulation of CRC cell colony formation induced by miR-130a-3p mimics (Figure 5g).

**Figure 5.** WNT1 overexpression reduces the suppressive effect of miR-130a-3p on c-myc and cyclin D1 expression. (a–f) CRC cells were co-transfected with a lentivirus WNT1 overexpression vector and miR-130a-3p mimic or mimic control. RT-qPCR and Western blot revealed that enhanced WNT1 expression attenuates the downregulation of c-myc and cyclin D1 induced by miR-130a-3p. (g) Results of CRC cell colony formation assay. **P < 0.01 vs. miR-mimics + pHAGE group. a. miR-mimics; b. miR-mimics+pHAGE; c. miR-mimics + pHAGE-wnt1. CRC, colorectal cancer

### MiR-130a-3p inhibits colorectal cancer cell growth in nude mice

We compared tumor growth among nude mouse groups injected subcutaneously with transfected HCT116 cells and HCT116 cells, aiming to further verity inhibition of CRC proliferation by miR-130a-3p. Tumors generated by CRC cells overexpressing miR-130a-3p mimics were significantly smaller as evidenced by lower weight and volume compared with tumors derived from control or mimic control cells (P < 0.01) (Figure 6a-c). In transplanted tumor tissue, in comparison with control groups, WNT1, Cyclin D1, and c-myc mRNA expression was decreased in mimics group (Figure 6d). Collectively, consistent result was get by *in vivo* experiment as by in *vitro* ones in determination of inhibition of CRC cell growth by miR-130a-3p overexpression.

**Figure 6.** Overexpressed miR-130a-3p inhibits colorectal cancer cell growth in a mouse xenograft model. (a-c) The total weights and volumes of tumors derived from the indicated CRC cell line were decreased by miR-130a-3p overexpression (mimics group) compared with control CRC cell lines. (d) RT-qPCR results showed WNT1, Cyclin D1 and c-myc mRNA expression was downregulated in mimics group, compared with control and mimics control groups. **P < 0.01. Per group n = 6

## Discussion

MiRNAs are multifunctional regulators of tumorigenesis and cancer progression, and miRNAs with tumor suppressor activities have been proposed as adjuvant therapies. These miRNAs, such as miRNA-506-3p, miRNA-143, miRNA-330, miR-141-3p, and miRNA-877 [19–23], inhibit tumorigenesis or progression by targeting oncogenic genes or signaling pathways. Both *in vitro and in vivo* experiments by Tian et al. reported the inhibition of migration and invasion by miR-130a-3p in esophageal squamous cell carcinoma cell line EC-1 [24]. miR-130a-3p also regulates Gemcitabine resistance via targeting PPARG in Cholangiocarcinoma [25]. Triple-negative breast cancer samples showed downregulated miR-130-3p in comparison with matched peritumoral tissues [26], and Wang et al. demonstrated the promotion of cervical cancer cell progression by miR-130a-3p was achieved by suppressing RUNX3 expression [27]. However, no study on effects of miR-130a-3p on CRC has been reported. We first analyzed the CRC samples from the TGCA database and found significantly reduced miR-130a-3p expression in comparison with normal tissue. Consistent result was got in our CRC tissues samples as in these bioinformatics results. Further, compared with the normal colon epithelial line NCM460, miR-130a-3p expression was reduced in multiple CRC cell lines (HCT116, SW480, LOVO, SW620, and HT29), and miR-130a-3p overexpression-induced promotion of CRC cell proliferation both *in vivo* and *in vitro*. Collectively, miR-130a-3p normally serves to inhibit CRC development.

The WNT signaling pathways influence malignancy by regulating cancer cell proliferation, differentiation, apoptosis, cell cycle progression, adhesion, and vascular regeneration [28–30]. It is believed that the key to WNT pathway-dependent carcinogenesis is the suppression of beta-catenin degradation, which causes the aggregation of free β-catenin in cytoplasm and its binding to Tcf/Lef transcription factors in the nucleus, thereby activating the transcription of oncogenic downstream target genes cyclin D1 and c-myc [31]. Poodineh et al. have been reported that miR-130a-3p could block the expression of Wnt signaling cascade gene (ZEB1, CTNNB1, LRP6, FZD6, Wnt2B) in breast cancer, and highly expressed miR-130a-3p could reduce migration and proliferation in triple-negative breast cancer [32]. This indicated miR-130a-3p acted as a regulator of Wnt/β -catenin cascade, however, its role in Wnt/β -catenin pathway is still of an unknown. In this study, TargetScan, RIRDB, and RIWALK predicted WNT1 targeting by miR-130a-3p, and its overexpression led to significant reduction in WNT1 expression at both mRNA and protein levels. Further, luciferase assays confirmed miR-130a-3p binding to the wild-type 3ʹUTR of WNT1 gene.

Cyclin D1, an oncogene, is one of the main factors regulating cell proliferation. Overexpression and upregulation of cyclin D1 are associated with abnormal cell cycle regulation and tumorigenesis [33]. Similarly, amplification or overexpression of c-myc gene can lead to the progression of colon cancer and other tumors [34]. Both cyclin D1 and c-myc are downstream targets of WNT1 pathway, strongly suggesting that downregulation by overexpressed miR-130a-3p involves the WNT1 pathway inhibition *in vivo and in vitro*. Consistent with this notion, overexpressed WNT1 reversed suppression of cyclin D1 and c-myc expression induced by miR-130a-3p. All of these indicate that miR-130a-3p targets WNT1 and regulates the development of CRC.

## Conclusion

This study demonstrates that miR-130-3p can suppress the proliferation of CRC cells both *in vitro* and *in vivo*, suggesting that miR-130-3p serves as an endogenous suppressor of CRC, possibly by downregulating WNT1 signaling and ensuing activation of oncogenic cyclin D1 and c-myc. Elucidation of the complete signaling pathway mediating the anti-cancer efficacy of miR-130-3p may identify novel therapeutic targets for CRC treatment.

## Data Availability

The data analyzed during the study is available from the corresponding author on reasonable request.

## Highlights

1. MiR-130a-3p is downregulated in colorectal cancer (CRC).
2. MiR-130a-3p overexpression inhibits CRC cell proliferation *in vitro* and *in vivo*.
3. MiR-130a-3p inhibits CRC growth by directly targeting WNT1.
